# Combined Application of Grid Body Surface Locator and Preemptive Analgesia in Daytime Vertebroplasty

**DOI:** 10.1155/2022/2651062

**Published:** 2022-07-25

**Authors:** Hongwen Gu, Yuhui Zhao, Yanchun Xie, Yongcun Wei, Linyang Li, Di Meng, Hailong Yu

**Affiliations:** ^1^Department of the Spine, General Hospital of Northern Theater Command, China; ^2^Dalian Medical University, Dalian, China; ^3^Panjin Liaoyou Gem Flower Hospital, Panjin, China; ^4^Jinzhou Medical University, Jinzhou, China

## Abstract

**Objective:**

To explore the clinical advantages of grid body surface locator combined with preemptive analgesia in the treatment of osteoporotic lumbar fractures in daytime vertebroplasty.

**Methods:**

A retrospective study was conducted on 120 patients who underwent lumbar vertebroplasty in the Department of Orthopedics of General Hospital of Northern Theater Command from January 2017 to January 2020. According to the preoperative planning and analgesic mode of treatment, they were divided into the daily operation experimental group and the traditional mode control group. Prone positioning of a patient under anesthetic is safe of ensuring optimum surgical access for many procedures, providing that the risks are fully understood. The general baseline data, intraoperative fluoroscopy times and operation time, bone cement injection volume, bone cement permeability, VAS score before operation, 1 day, and 3 months after operation, and the recovery of anterior vertebral height before and after operation were analyzed.

**Results:**

There was no statistically significant difference in the preoperative general data between the two groups. One day after operation, the VAS score of the experimental group was lower than that of the control group, but there was no difference after 3 months. The permeability of bone cement in the experimental group was lower than that in the control group, the height of anterior edge of injured vertebra was better than that in the control group, and the operation time was less than that in the control group.

**Conclusion:**

The daytime operation experimental group can significantly alleviate postoperative pain, increase the amount of bone cement injection, and reduce the permeability of bone cement through preoperative planning of puncture path and key puncture points, combined with advanced labor pain, but there is no significant difference in long-term pain relief.

## 1. Introduction

With the aging of the population, the problem of osteoporosis is becoming more and more prominent, followed by an increase in the number of vertebral fracture groups [1–3]. At present, vertebroplasty is an effective and commonly surgical treatment for osteoporotic vertebral compression fractures [4–6]. Vertebroplasty is a minimally invasive surgery that injects bone cement into the injured vertebra through the puncture channel for pain relief and high reduction [7]. During the vertebroplasty operation, a needle is percutaneously inserted into the fractured vertebra, and bone cement is injected to stabilize the fracture site [8]. The vertebral body is adjacent to important blood vessels and nerves, so the accuracy of puncture is particularly important. Vertebroplasty has been proven as an effective treatment for osteoporotic vertebral compression fractures, with a high success rate and relatively less complications. However, bone cement leakage has been reported as a main concern in previous studies. This leakage could enter the spinal cavity, intervertebral foramen, vertebral vein, and inferior vena cava via channels caused by the trauma, leading to severe local or systemic complications, or even death. Because puncture is aimed at soft tissue injury, intraoperative and postoperative pain may be aggravated [9, 10]. In particular, some fractured people have a sense of fear and pain about the operation.

The prone position under local anesthesia takes a long time during the operation, resulting in resistance, which cannot be well-matched with the operation. Prone positioning of a patient under anesthetic is safe of ensuring optimum surgical access for many procedures, providing that the risks are fully understood. In serious cases, it will also lead to operation failure [11, 12]. Therefore, this study focuses on puncture and analgesia during vertebroplasty and carries out relevant research to reduce the operation time, reduce patients' pain, and ensure the safety of operation.

## 2. Data and Methods

As reported in the criteria for the appropriate treatment of osteoporotic vertebral compression fractures [13], the inclusion and exclusion criteria are as follows.

### 2.1. Inclusion Criteria

The following are the inclusion criteria: (1) osteoporotic vertebral compression fracture, (2) no neurological symptoms, and (3) the injured vertebrae were single-segment lumbar vertebrae.

### 2.2. Exclusion Criteria

The following are the exclusion criteria: (1) received lumbar surgery and (2) tumor, infection, and other diseases.

### 2.3. General Data

A retrospective analysis of 120 cases who underwent lumbar vertebroplasty in the Department of Orthopedics of our hospital from January 2017 to January 2020 was carried out. According to the preoperative planning and analgesic mode of treatment, they were divided into the daily operation experimental group and the traditional mode control group. All cases were operated by the same experienced spine surgeon through unilateral puncture, and the bone mineral density (*t* value) was measured by dual-energy X-ray (DXA) before operation. There were 60 cases in the traditional mode control group, 40 males and 20 females, aged 55-84 years, with an average age of 75.109 ± 2.198 years, and the average preoperative *t* value was −2.221 ± 0.574. There were 60 cases in the daily operation experimental group, 36 males and 24 females, aged 59-82 years, with an average age of 72.342 ± 3.342 years, and the preoperative average *t* value was −2.191 ± 0.434. See Table 1 for details.

### 2.4. Operation Process

#### 2.4.1. Operation Process of the Traditional Mode Control Group

Lie prone during operation, local anesthesia, select “9 points” (left side) or “3 points” (right side) of the projection of the pedicle of the fractured vertebral body as the needle entry point under fluoroscopy, and when the puncture needle tip reaches the inner edge of the pedicle and the lateral position is at the posterior edge of the vertebral body, it is the “safe position,” and continue to enter the puncture needle for about 0.5 cm, which was dedicated to the monitoring and recording of vital parameters, such as body temperature, heart rate and rhythm, respiration, oxygen saturation via pulse oximetry, blood pressure, and end-tidal carbon dioxide. After the puncture, insert the guidewire and working channel and inject bone cement.

#### 2.4.2. The Control of the Puncture Angle

The angle of the needle at point B is determined by the protractor (angle ABC). With this available data, the distance from point B (on the skin surface) to point C (the target calyx) is calculated using the law of Sines. This is easily done by the Universal Triangle Solver application on Google Play® (easily downloaded on any smart phone). Herein, if we have two angles and one side of a triangle, then we can calculate the other angle and sides. For example, if the angle ABC, i.e., the angle at the point B, is 65°, the distance AB is 4 cm, and the angle CAB is always 90°, then, by the Universal Triangle Solver, we have the distance B to C calculated as 9.5 cm, which is the depth of puncture. Thus, the depth and angle of puncture are estimated using the bull's eye technique.

#### 2.4.3. Operation Process of the Daily Operation Experimental Group

The patient is prone, the grid body surface locator is placed on the body surface, and the CT scanning of the fractured vertebral body and body surface grid locator is carried out to achieve the purpose of skin data visualization (Figure 1). The CT data is imported into Mimics software to build the weight of the fractured vertebral body and plan the puncture path.

Anesthesia and position (step 1): this study believes that the three key points to complete the unilateral puncture path include the skin puncture point (point A), vertebral bone puncture point (point B), and intravertebral landing point (point C). The location of point C designed in this study: horizontal plane: the midpoint of the connecting line between the upper and lower endplates of the vertebral body; sagittal plane: the anterior third of the centrum; point B is the midpoint of the pedicle. After connecting point C and point B, make a reverse extension line and the intersection with the skin is point A. The position of point a can be determined by the grid body surface locator placed before operation (Figure 2). Approach and exposure (step 2): mark the skin puncture point with a marker pen, evenly apply about 1 g of compound lidocaine cream around the mark point 1 hour before operation, and seal the dressing on the upper cover. Half an hour before operation, 50 mg was given intravenously. During operation, 5 ml: 0.1 g lidocaine hydrochloride injection and 0.1% mixed normal saline were diluted to 20 ml, and local anesthesia was performed along the preoperative planning trajectory of Mimics software. Finally, the puncture needle was inserted and bone cement was injected along the trajectory Figure 3.

### 2.5. The Visual Analogue Scale

The visual analogue scale (VAS) is commonly used as the outcome measure for such studies. It is usually presented as a 100 mm horizontal line on which the patient's pain intensity is represented by a point between the extremes of “no pain at all” and “worst pain imaginable.”

### 2.6. Statistical Analysis

Statistical analysis was performed by SPSS 22.0 (SPSS Company, USA) statistical software package. The measurement data were expressed by ($\overset{¯}{x}\pm s$). The statistical analysis was performed by comparative *t*-test (*P* < 0.05 statistical significance). The general baseline data, intraoperative fluoroscopy times, operation time, bone cement injection volume, bone cement permeability, VAS score before operation, 1 day after operation, and 3 months after operation were analyzed and compared the recovery of anterior vertebral height before and after operation.

## 3. Results

There was no significant difference in preoperative age, sex, bone mineral density (*t* value), and fracture distribution between the two groups (see Table 1). As shown in Table 2, VAS score 1 day after operation of daily operation experimental group (3.312 ± 0.421) was higher than the traditional mode control group (2.563 ± 0.574). But no statistical significance was found in preoperative VAS score or VAS score 3 months after operation, which indicated that permeability of bone cement in the experimental group was lower than that in the control group. The VAS scores of the two groups were significantly improved one day and three months after operation, and the VAS of the experimental group was significantly lower than that of the control group one day after operation, but there was no significant difference between the two groups three months after operation. Three months after operation, the anterior edge of vertebral body (ah) of the two groups was improved, and the experimental group was better than the control group.

For the sake of height of anterior edge of injured vertebra, the daily operation experimental group (21.236 ± 1.489) was better than the traditional mode control group (22.149 ± 1.389). The operation time of daily operation experimental group (24.253 ± 2.873) was lower than that in the control group (28.833 ± 4.317).

The number of intraoperative positioning fluoroscopy, total fluoroscopy, and operation time in the daytime operation experimental group was significantly lower than those in the traditional mode control group, and the amount of bone cement injection was significantly higher than that in the control group (see Table 2).

After preoperative planning and body surface grid positioning, the results show that the bone cement is fully healed (Figure 4). And the patients were followed up for 1 year after operation with coronal, sagittal, and axial CT and the bone cement was fully diffused (Figure 3).

## 4. Discussion

Day surgery is a kind of surgery mode that is hospitalized on the same day and operated on and discharged within 24 hours, also known as nonhospitalized surgery [13]. For osteoporotic vertebral compression fractures of the spine, vertebroplasty is a relatively simple and effective minimally invasive treatment [14, 15]. Surgeons have the problem that the puncture positioning process is not accurate enough to puncture many times, which causes great psychological pressure, especially for junior doctors [16]. Considering the current problems of vertebroplasty, this study carried out a new daytime operation mode through channel planning, skin epidermal anesthesia with local compound lidocaine cream before operation, advanced anesthesia with intravenous infusion of flurbiprofen axetil injection, and multimodal analgesia combined with local infiltration anesthesia of intraoperative lidocaine injection, to realize rapid and slight pain of vertebroplasty safe surgical treatment. The grid body surface locator of this study, as previously reported [17–19], can rely on CT data to reconstruct the injured vertebra and body surface grid locator before vertebroplasty and realize “one-time” placement of the puncture channel according to the planned path and angle. Fewer puncture times and adjustment of puncture needle position can not only avoid pain but also reduce puncture failure and bone cement leakage. The robots are convenient in helping deciding the position and treatment methods for patients, and the wound will be thin. The robots are expensive. Given the high price of robots, body surface locator is an effective positioning method that can be popularized in a large range. Moreover, accurate body surface positioning can be implemented according to the body surface grid device. When applying compound lidocaine cream on the skin, epidermal anesthesia can effectively reduce the scope and reduce the harm of local reactions such as pallor, erythema and edema, and allergic reactions. This is the complementarity of “positioning” and “intoxication” [20, 21].

Before the operation, compound lidocaine cream was applied, and flurbiprofen axetil injection was injected intravenously for preemptive analgesia according to the half-life of the drug. Compound lidocaine cream contains lidocaine and procaine. Lidocaine is a short-acting local anesthetic with fast onset; procaine has a long duration of efficacy and is the drug with the longest duration of efficacy in local anesthetics [22]. Therefore, compound lidocaine cream has the characteristics of fast onset and long maintenance time. Compared with the puncture method using a “clock point” in the traditional model, using the grid body surface locator to plan the puncture point, path and angle are more accurate, significantly reduce the puncture time, fully diffuse the bone cement, and then significantly reduce the bone cement permeability [17–19]. The puncture channel planned for daytime surgery is completely located in the bone structure, and the puncture midpoint is located in the middle third of the anterior part of the vertebral body, far from the vertebral basal venous plexus. It is a low incidence area of bone cement leakage. At the same time, the central area can maximize the diffusion of bone cement. Bone cement filling can effectively increase the strength and stiffness of vertebral body, alleviate the pain of vertebral fracture, restore the height of vertebral body, and increase the ability to bear stress [23]. When bone cement contacts one side of the surface of the upper and lower endplates, the stiffness and strength can be increased by 3 times. When contacting the upper and lower endplates at the same time, it can be increased by 11 times [24]. The puncture path planning is located in the center of the injured vertebra, which is conducive to the uniform dispersion of bone cement. It is more likely to contact the upper and lower endplates before leakage, which is more conducive to the effect after operation. Therefore, compared with the traditional model control group, the safety and efficacy of daytime surgery have been significantly improved.

Limitations of this study are as follows: this study is a preliminary exploration under daytime vertebroplasty, and the number of control cases is small. There may be a small error when the patient completes CT shooting in the imaging department and enters the operating room for repositioning. Only a single osteoporotic compression fracture of the lumbar spine was studied, and multiple fractures, thoracic fractures, and Kummell disease were not considered.

## 5. Conclusion

To sum up, considering the current problems of vertebroplasty, this study uses a grid body surface locator for channel planning, combined with preemptive analgesia and other means to carry out new daytime surgery, so as to achieve rapid, slightly painful, and safe treatment of osteoporotic vertebral fractures.

## Figures and Tables

**Figure 1:** (a) Schematic diagram and grid display of grid body surface locator. (b) Schematic diagram of grid body surface locator placed on body surface. (c) Schematic diagram of CT scanning of grid body surface locator placed on body surface.

**Figure 2:** Observation of injured vertebrae, puncture site, and puncture path planning of mimics reconstruction from different angles ((a) sagittal position, (b) coronal position, and (c) frontal position).

**Figure 3:** The patients were followed up for 1 year after operation with coronal, sagittal, and axial CT and the bone cement was fully diffused.

**Figure 4:** Puncture site, path planning, and sufficient and uniform dispersion of bone cement (the patient is a 60-year-old female with osteoporosis lumbar fracture). After preoperative planning and body surface grid positioning, it can be seen that the bone cement is fully healed.

**Table 1:** Comparison of preoperative general baseline data between the two groups.

Group	Daily operation experimental group	Traditional mode control group	*P*
*N*	60	60	—
Age	72.342 ± 3.342	75.109 ± 2.198	0.243
Gender (male/female)	36/24	40/20	0.126
Average *t* value	−2.191 ± 0.434	−2.221 ± 0.574	0.271
Fracture vertebral body distribution			0.344
L1	30	32	
L2	19	18	
L3	7	8	
L4	3	2	
L5	1	0	

**Table 2:** Comparison of intraoperative conditions, preoperative and postoperative VAS, and anterior height of injured vertebrae between the two groups.

Group	Daily operation experimental group	The traditional mode control group	*P*
*n*	60	60	—
Positioning perspective times (times)	15.733 ± 2.492	7.627 ± 1.668^∗^	0.006
Total fluoroscopy times (times)	26.200 ± 4.313	20.867 ± 2.924^∗^	0.018
Operation time (min)	24.253 ± 2.873	28.833 ± 4.317^∗^	<0.001
Bone cement injection volume (ml)	4.519 ± 1.269	6.319 ± 1.648^∗^	<0.001
Preoperative VAS score (score)	8.102 ± 0.587	7.802 ± 0.431	0.148
VAS score 1 day after operation (score)	3.312 ± 0.421	2.563 ± 0.574	<0.001
VAS score 3 months after operation (score)	1.781 ± 0.241	1.801 ± 0.385	0.351
Height of anterior edge of injured vertebra before operation (mm)	17.733 ± 2.492	17.267 ± 2.668	0.118
Height of anterior edge of injured vertebra 3 months after operation (mm)	21.236 ± 1.489^∗^	22.149 ± 1.389^∗^	0.021

## Data Availability

The data could be obtained by contacting the corresponding author.
